# Rpb3 promotes hepatocellular carcinoma through its N-terminus

This article has been retracted.

**DOI:** 10.18632/oncotarget.2389

**Published:** 2014-09-02

**Authors:** Zhe-Ping Fang, Bei-Ge Jiang, Fa-Biao Zhang, Ai-Dong Wang, Yi-Ming Ji, Yong-Fu Xu, Ji-Cheng Li, Wei-Ping Zhou, Wei-Jie Zhou, Hai-Xiong Han

**Affiliations:** ^1^ Department of Hepatobiliary Surgery, Taizhou Hospital of Zhejiang Province, Wenzhou Medical University, Linhai 317000, China; ^2^ Eastern Hepatobiliary Surgery Hospital, Second Military Medical University, Shanghai 200438, China; ^3^ Institute of Cell Biology, Zhejiang University, 866 Yu-Hang-Tang Road, Hangzhou 310058, China; ^4^ Department of Biologic and Materials Sciences, University of Michigan School of Dentistry, Ann Arbor, MI 48109, USA

**Keywords:** Hepatocellular carcinoma, liver tumorigenesis, Proliferation, Rpb3

## Abstract

The expression of RNA polymerase II subunit 3 (Rpb3) was found frequent up-regulation in Hepatocellular carcinoma (HCC) tumors. Significant associations could also be drawn between increased expressions of Rpb3 and advance HCC staging and shorter disease-free survival of patients. Overexpression of Rpb3 increased HCC cell proliferation, migratory rate and tumor growth in nude mice, whereas suppression of Rpb3 using shRNA inhibited these effects. For mechanism study, we found that Rpb3 bound directly to Snail, downregulated E-cadherin, induced HCC cells epithelial-mesenchymal transition (EMT). In particular, N-terminus of Rpb3 blocked Rpb3 binding to Snail, inhibited Rpb3-high-expression HCC cells proliferation, migration, tumor growth in nude mice, and also inhibited DEN-induced liver tumorigenesis. Furthermore, N-terminus of Rpb3 did not inhibit normal liver cells or Rpb3-low-expression HCC cells proliferation. These findings suggest that N-terminus of Rpb3 selectively inhibits Rpb3-high-expression HCC cells proliferation. N-terminus of Rpb3 may be useful in treating patients diagnosed with Rpb3-high-expression HCC.

## INTRODUCTION

Hepatocellular carcinoma (HCC) is the fifth most common solid tumor worldwide and the third leading fetal cancer [1]. In spite of significant technical improvements in curative treatments such as surgical resection and transplantation, the prognosis of patients with HCC remains very poor due to invasion and metastasis. For development of targeted therapies with positive results, it is important to understand the molecular characteristic and related biological mechanism in HCC cell proliferation, migration and metastasis.

In eukaryotes, three RNA polymerases play fundamental roles in the cell. RNA polymerase I and III transcribe ribosomal DNA, tRNAs and small nuclear RNA genes. RNA Pol II transcribes protein coding genes and some small nuclear RNA genes [2]. This enzyme consists of 12 different subunits and is subjected to many controls, including initiation, elongation and termination of mRNA transcription.[3] However, little is known about the specific functions of its individual subunits, associations between subunits, or possible contacts between subunits and transcription factors. Rpb11 and Rpb3 have been shown involvement in doxorubicin (dox)-mediated cellular toxicity and cellular differentiation [4, 5]. In myoblast cells, Rpb3 expression is regulated during cell differentiation, it binds to myogenic factor, ATF4 and IGF-binding protein (IGFBP)-3, and increases their transactivation activity [6-8]. Eukaryotic translation elongation factor 1 gamma (eEF1γ) is identified as another Rpb3 binding partner, which binds to Vimentin promoter [9]. It would be very interesting to explore the roles of individual subunits besides their function in RNA polymerases complex.

The Snail family members Snail and Slug are essential for triggering EMT during embryonic development and tumor progression [10-13]. In the current study, we reported for the first time that Rpb3 played as an oncogene in HCC. We identified Rpb3 as a new Snail binding partner. We found that N-terminus of Rpb3 inhibited Rpb3-high-expression HCC cells proliferation, migration, tumor growth, and liver tumorigenesis.

## RESULTS

### Rpb3 is frequently up-regulated in HCC and correlates with progressed HCC and shortened survival

We first detected the expression of Rpb3 protein in human HCC samples using immunohistochemical analysis. Using an antibody for Rpb3 staining, we examined tissue samples from 322 patients with a pathological diagnosis of HCC. Up-regulated Immunoreactivity for the Rpb3 antigens was observed in 16.13% (5/31) of the patients with Stage I HCC tissues, 36.67% (33/90) of the patients with Stage II HCC tissues, 54.72% (58/106) the patients with Stage III HCC tissues, and 72.63% (69/95) the patients with Stage IV HCC tissues. Notably, the staining of Rpb3 was much stronger in high-grade HCC than in low-grade HCC (Fig. 1A and 1B). To confirm the up-regulation of Rpb3, real-time qPCR analysis was performed using 322 normal liver adjacent tissue samples and 322 HCC tissue samples. Consistent with the results of the immunohistochemical analysis, advanced stage of HCC expressed higher Rpb3 mRNA (Fig. 1C). Rpb3 mRNA levels also were shown positively associated with the histologic presence of micro-vascular invasion (Fig. 1D). We also detected the expression of other subunits of the RNA Pol II, including the two largest subunits Rpb1 and Rpb2, which form the catalytic core of the enzyme, and Rpb3 directly binding subunits Rpb11. None of Rpb1, Rpb2 or Rpb4-12 expression was observed up-regulated in HCC samples (Supplemental Figure S1, A-K).

**Figure 1:** Clinicopathologic correlation of Rpb3 expression in HCC **(A)** Representative images for the expression level of Rpb3 in normal tissue compared with stage I-IV HCC tissues detected through immunostaining with the Rpb3 antibody. Bar = 50 μm. **(B)** A positive percentage of Rpb3 expression in stage I-IV HCC. **(C)** The expression of Rpb3 was verified through real-time qPCR in normal tissues and HCC samples. Each box represents the 5th and 95th percentiles, the middle line represents the mean value, and the whiskers represent the standard deviation. **(D)** Elevated STK33 expression showed marked association with tumors baring microvascular invasion. **(E, F)** Kaplan-Meier analyses were performed according to Rpb3 mRNA expression in HCC patients. The overall survival of patients with positive Rpb3 expression was evidently shorter **(E)**. The disease-free survival of patients with positive Rpb3 expression was evidently shorter **(F)**. Kaplan-Meier analyses were performed according to Rpb3 protein expression scores in HCC patients. Immunostaining score 0-2 and ≥3 were considered to indicate negative and positive expression of Rpb3, respectively. The results represent at least three separate experiments. Error bar, ± S.D. * *p* < 0.05, ** *p* < 0.01.

We further evaluated whether the Rpb3 expression correlated with overall survival in 322 patients with HCC. We observed that the up-regulation of Rpb3 predicted shorter overall survival and the disease-free survival of HCC patients (Fig. 1E and 1F). The multivariate survival analysis using the Cox proportional hazards model further indicated that the up-regulation of Rpb3 was correlated with a higher hazard ratio (HR) and poor clinical outcomes (overall survival, *p* = 0.005, HR 4.638; for disease-free survival, *p* = 0.016, HR 2.986) (Table 1, the main features of the patients in this study could be find in Supplemental Table1). These results highlight the clinical importance of Rpb3 in determining the prognosis for patients with HCC, indicating a new target for HCC therapy.

**Table 1:** Multivariate cox regression analysis of Rpb3 expression in HCC

Varable	Overall Survival		Disease-Free Survival	
	HR (95% CI)	*p* Value	HR (95% CI)	*p* Value
Rpb3 expression	4.623 (1.633-8.465)	**0.008**	2.986 (1.267-5.832)	**0.022**
Sex	0.746 (0.165-3.298)	0.669	0.803 (0.208-2.391)	0.413
Cirrhosis*	1.966 (0.603-5.935)	0.260	1.223 (0.478-2.531)	0.625
HBsAg**	4.085 (0.529-34.192)	0.188	1.230 (0.327-3.135)	0.762
Microvascular invation	2.823 (0.449-6.013)	**0.012**	2.309 (0.220-3.780)	0.062
Clinical stage***	3.722(0.665-12.369)	**0.028**	2.884 (0.537-6.025)	**0.032**

Abbreviations: CI, confidence interval; HBsAg, Hepatitis B surface antigen; HR, hazard ratio.

Boldface highlights the statistical significance.

* Presence versus absence.

** Hepatitis B virus positive versus negative

*** Early (T1/T2) versus advanced stage (T3/T4).

### Rpb3 enhances HCC cells growth and migration

We next examined the expression of Rpb3 in HCC cell lines using anti-Rpb3 antibodies using western blotting. Compared with normal liver tissue lysate, elevated Rpb3 expression was observed in 5 of the 6 HCC cell lines, These results were also confirmed through real-time qPCR analysis (Supplemental Figure S2, A and B). However, the expression of all other subunits of RNA Pol II, Rpb1, Rpb2 and Rpb4-12, was not observed up-regulated in these HCC cell lines (Supplemental Figure S2, C-M).

To investigate the biological role of Rpb3 in HCC cells, we performed gain- or loss-of-function studies. We overexpressed Rpb3 in QGY-7701 cells and HepG2 cells, which expressing lower endogenous Rpb3 (Fig. 2A). We subsequently examined the role of Rpb3 in HCC cell proliferation using MTT assay and BrdU assay. The results indicated that cell proliferation was enhanced *in vitro* after transfection with Rpb3 in both QGY-7701 and HepG2 cells (Fig. 2B and 2C). Using boydon chamber cells migration assay, more migrated cells were found in Rpb3-overexpressing QGY-7701 cells and HepG2 cells (Fig. 2D). We then examined whether Rpb3 enhanced tumor growth *in vivo*. When cells were injected subcutaneously into athymic nude mice, the overexpression of Rpb3 resulted in dramatically increased tumor volumes compared with the vector controls for both QGY-7701 and HepG2 cells *in vivo* (Fig. 2E).

**Figure 2:** Rpb3 promotes HCC cell proliferation, migration and *in vivo* tumor growth **(A)** QGY-7701 and HepG2 cells transfected with plain vector (V) or plasmid encoding Rpb3 (Rpb3). Cell lysates were immunoblotted using the Rpb3 antibody, actin was used as the loading control. **(B)** *In vitro* growth of QGY-7701/V, HepG2/V (V) and QGY-7701/Rpb3, HepG2/Rpb3 (Rpb3) cells, measured using MTT assay. **(C)** *In vitro* growth of QGY-7701/V, HepG2/V (V) and QGY-7701/Rpb3, HepG2/Rpb3 (Rpb3) cells measured using BrdU assays. **(D)** Migrated cells numbers of QGY-7701/V, HepG2/V (V) and QGY-7701/Rpb3, HepG2/Rpb3 (Rpb3) cells were counted. **(E)** Average tumor volume in athymic nude mice subcutaneously inoculated with QGY-7701/V, HepG2/V (V) and QGY-7701/Rpb3, HepG2/Rpb3 (Rpb3) cells. **(F)** HCC-LM3 and SMMC7721 Cells transfected with control shRNA (Ctrl shRNA) or Rpb3 shRNA1 and Rpb3 shRNA2. Rpb3 levels were detected through immunostaining using Rpb3 antibody, with actin as the loading control. **(G, H)** *In vitro* growth of HCC-LM3/Control shRNA and SMMC-7721/Control shRNA (Ctrl shRNA), HCC-LM3/Rpb3 shRNA1 and SMMC-7721/Rpb3 shRNA1 (Rpb3 shRNA1) cells, HCC-LM3/Rpb3 shRNA2 and SMMC-7721/Rpb3 shRNA2 (Rpb3 shRNA2) cells, measured using MTT assay (G) and BrdU assay (H). **(I)** Migrated cells numbers were counted when HCC-LM3 and SMMC-7721 cells were treated with control shRNA (Ctrl shRNA), Rpb3 shRNA1 and Rpb3 shRNA2. **(J)** Average tumor volume in athymic nude mice subcutaneously inoculated with HCC-LM3/Control shRNA and SMMC-7721/Control shRNA (Ctrl shRNA), HCC-LM3/Rpb3 shRNA1 and SMMC-7721/Rpb3 shRNA1 (Rpb3 shRNA1) cells, HCC-LM3/Rpb3 shRNA2 and SMMC-7721/Rpb3 shRNA2 (Rpb3 shRNA2) cells. For (A, B, C, E, F, G), the results represent at least three separate experiments. For (D and H), n=10 mice/group. Error bar ± S.D. * *p* < 0.05, ** *p* < 0.01.

To further investigate the function of Rpb3 in HCC cell proliferation, migration and tumor growth, we used Rpb3 shRNA to knockdown Rpb3 expression in both HCC-LM3 and SMMC-7721 cells, which both expressed abundant endogenous Rpb3 protein (Fig. 2F). Compared with control shRNA (Ctrl shRNA), the cells treated with Rpb3 shRNA1 and Rpb3 shRNA2 grew more slowly *in vitro* (as determined through MTT assay and BrdU assay) in both HCC-LM3 and SMMC-7721 cells (Fig. 2G and 2H). The migrated cells numbers of both HCC-LM3 and SMMC-7721 cells treated with Rpb3 shRNAs also decreased (Fig. 2I). The mice inoculated subcutaneously with HCC-LM3/Rpb3 shRNA1 cells, HCC-LM3/Rpb3 shRNA2 cells and SMMC-7721/Rpb3 shRNA1 cells, SMMC7721/Rpb3 shRNA2 cells, exhibited dramatically reduced tumor volumes compared with mice receiving HCC-LM3/Ctrl shRNA and SMMC-7721/Ctrl shRNA cells (Fig. 2J). These *in vitro* and *in vivo* results demonstrate that Rpb3 potently promotes HCC cells proliferation, migration and tumor growth.

### Rpb3 promotes HCC cells EMT induction and inhibits E-cadherin transcription

Given that up-regulated Rpb3 correlated with enhanced cell migratory abilities of HCC cells, we nest examined the EMT as an underlying mechanism. In QGY-7701 and HepG2 cells, overexpression of Rpb3 down-regulated epithelial markers E-cadherin, Claudin1 and ZO-1, and up-regulated mesenchymal markers N-cadherin and Vimentin. In HCC-LM3 and SMMC-7721 cells, Rpb3 shRNA up-regulated epithelial markers E-cadherin, Claudin1 and ZO-1, and down-regulated mesenchymal markers N-cadherin and Vimentin (Fig. 3A). We also detected HCC samples for EMT marker expression using qRT-PCR assay, we found that Rpb3 positive HCC sample showed less mRNA expression of epithelial markers and more mRNA expression of mesenchymal markers (Fig. 3B).

**Figure 3:** Rpb3 induces HCC cells EMT, inhibits E-cadherin transcription **(A)** Western blots show a significant decrease in expression of epithelial markers E-cadherin, Claudin1 and ZO-1 and a corresponding increase in the levels of the mesenchymal markers N-cadherin and Vimentin in QGY-7701 and HepG2 cells when Rpb3 was over-expressed. Knockdown of Rpb3 in HCC-LM3 and SMMC-7721 cells induced significant increase in expression of epithelial markers E-cadherin, Claudin1 and ZO-1 and a corresponding decrease in the levels of the mesenchymal markers N-cadherin and Vimentin. **(B)** Western blots show a significant decrease in expression of epithelial markers E-cadherin, Claudin1 and ZO-1 and a corresponding increase in the levels of the mesenchymal markers N-cadherin and Vimentin in Rpb3 positive HCC samples compared to Rpb3 negative HCC samples (n=150/group). **(C)** Rpb3 overexpression decreased mRNA level of E-cadherin in HepG2 cells. **(D)** Rpb3 knockdown increased mRNA level of E-cadherin in HCC-LM3 cells. **(E)** Rpb3 overexpression decreased E-cadherin promoter transcription in HepG2 cells. **(F)** Rpb3 knockdown increased E-cadherin promoter transcription in HCC-LM3 cells. The results represent at least three separate experiments. Error bar represent ± S.D. * *p* < 0.05.

E-cadherin is the most important molecular in promoting EMT induction, we next investigated whether Rpb3 regulated E-cadherin transcription. Using qRT-PCR assay, we found that overexpression of Rpb3 inhibited the mRNA level of E-cadherin in HepG2 cells (Fig. 3C), whereas knockdown of Rpb3 enhanced the mRNA level of E-cadherin in HCC-LM3 cells (Fig. 3D). To confirm that Rpb3 regulated E-cadherin transcription, we used E-cadherin promoter luciferase reporter assay, and found that overexpression of Rpb3 inhibited E-cadherin promoter transcription in HepG2 cells (Fig. 3E), whereas knockdown of Rpb3 enhanced E-cadherin promoter transcription in HCC-LM3 cells (Fig. 3F).

Snail is the key regulator to inhibit E-cadherin transcription, we next investigated whether Rpb3 regulated Snail induced E-cadherin transcription inhibition. Using E-cadherin promoter luciferase reporter assay, we found that Rpb3 facilitated further E-cadherin transcription inhibition induced by Snail (Supplemental Figure S3, A), and Snail failed to inhibit E-cadherin transcription when Rpb3 was knockdown using shRNA (Supplemental Figure S3, B). However, the endogenous Snail protein level was not changed by Rpb3 Supplemental Figure S3, C). These results indicated that association with Rpb3 is necessary for Snail to inhibit E-cadherin transcription.

### N-terminus of Rpb3 binds directly to Snail

We next explored the mechanism that how Rpb3 regulated Snail regulated E-cadherin transcription. Using co-immunoprecipitation (co-IP) assay in primary HCC samples lysates, we found that Snail could co-immunoprecipitated with endogenous Rpb3 (Fig. 4A). In HCC-LM3 cells, we also found that Snail could co-immunoprecipitated with endogenous Rpb3 (Fig. 4B). The binding between Rpb3 and Snail was further confirmed using IF assay, Rpb3 and Snail co-localizated in nucleus (Fig. 4C). We next examined whether Rpb3 interacted with Snail directly using purified recombinant proteins. A His tag was fused to the full length Snail (Snail-His), and a GST tag was fused to full length Rpb3 (Rpb3-F), N-terminus (aa1-160, Rpb3-N) or C-terminus (aa161-275, Rpb3-C, Fig. 4D). The N-terminus of Rpb3 but not the C-terminus bound directly to Snail-His (Fig. 4E). To further map the binding domain between Robo3 and Snail, we divided N-terminus of Rpb3 into three fragments: GST-Rpb3-N1 (aa1-50), GST-Rpb3-N2 (aa51-105), and GST-Rpb3-N3 (aa106-160, Fig. 4D). Through pull down assay, we found that the first 50 amino acid of Rpb3 is the necessary Snail binding domain (Fig. 4F).

**Figure 4:** Rpb3 binds directly to Snail and N-terminus of Rpb3 blocks Rpb3/Snail association **(A)** Endogenous Rpb3 bound to Snail in HCC samples. Endogenous Rpb3 was immunoprecipitated from the HCC tumor lysates using rabbit anti-Rpb3 antibody, followed by immunoblotting with antibodies to Rpb3 and Snail. Rabbit IgG (rIgG) was used as an immunoprecipitation negative control antibody. Sample loading controls are shown (2% input). **(B)** Endogenous Rpb3 bound to Snail in HCC-LM3 cells. Endogenous Rpb3 was immunoprecipitated from the cell lysates using rabbit anti-Rpb3 antibody, followed by immunoblotting with antibodies to Rpb3 and Snail. Rabbit IgG (rIgG) was used as an immunoprecipitation negative control antibody. Sample loading controls are shown (2% input). **(C)** Rpb3 (in red) and Snail (in green) colocalization was confirmed by immunofluorescence staining. Nuclei were counterstained with DAPI (in blue). Scale bar: 50μm. **(D)** Schematic illustration of Snail and Rpb3 mutants constructs. **(E** and **F)** Snail directly binds to N-terminus of Rpb3. Isolated His fused full length Snail protein (Snail-His), and GST fused full length Rpb3 protein (Rpb3-F), N-terminus of Rpb3 protein (Rpb3-N), C-terminus of Rpb3 protein (Rpb3-C), three mutants of N-terminus of Rpb3: Rpb3-N1, Rpb3-N2 and Rpb3-N3, were incubated with glutathione beads as indicated. After extensive washing, they were immunoblotted with the anti-His antibody for Snail detection; Rpb3 mutants were detected using anti-GST antibody. Sample loading controls are shown (2% input). Panel E showed Snail-His bound directly to Rpb3-F and Rpb3-N, and panel F showed His-Nail bound directly to Rpb3-N1. **(G)** Rpb3-N1 blocked endogenous Rpb3/Snail association. Adenovirus coding N-terminus of Snail (aa1-50, Ad-Rpb3-N1) and control vector (Ad-V) were infected into HCC-LM3 cells, Snail was immunoprecipitated from the cell lysates using rabbit anti-Snail antibody, followed by immunoblotting with anti-Rpb3 antibody for endogenous Rpb3 detection, anti-Snail antibody for endogenous Snail detection, and anti-Flag antibody for Rpb3-N1 mutant detection. Sample loading controls are shown (2% input). **(H)** Ad-Rpb3-N1 infection increased E-cadherin protein level in HCC-LM3 cells. **(I)** Ad-Rpb3-N1 infection increased E-cadherin promoter transcription in HCC-LM3 cells.

To test whether N-terminus of Rpb3 completed and blocked the Rpb3/Snail association, we developed adenovirus coding N-terminus of Snail (aa1-50, Ad-Rpb3-N1) fused with a Flag tag. We infected HCC-LM3 cells with adenovirus coding control vector (Ad-V) or Ad-Rpb3-N1, and got the stable cell lines. Through co-IP assay using antibody to Snail, we found that less endogenous Rpb3 co-immunopricipatitated with Snail when cells treated with Ad-Rpb3-N1, while Rpb3-N1 competed against endogenous Rpb3 to binding to Snail (Fig. 4G). We next explored whether Ad-Rpb3-N1 affected E-cadherin transcription. In fact, Ad-Rpb3-N1, but not Ad-V, increased both E-cadherin protein expression (Fig. 4H) and E-cadherin promoter transcription (Fig. 4I).

### N-terminus of Rpb3 inhibits HCC cells proliferation, migration and tumorigenesis

For studying the function of Rpb3-N1in HCC cells, we used MTT assay and BrdU assay, found that the proliferation ability of HCC-LM3 cells was dramatically inhibited by Ad-Rpb3-N1, but not by Ad-V, (Fig. 5A). Ad-Rpb3-N1 also inhibited HCC-LM3 cells migratory activity (Fig. 5B). Nude mice inoculated subcutaneously with HCC-LM3 cells treated with Ad-Rpb3-N1 had dramatically reduced tumor volumes compared with cells treated with Ad-V (Fig. 5C). The proliferation of SMMC-7721 cells was inhibited by Ad-Rpb3-N1 too (data not shown).

**Figure 5:** N-terminus of Rpb3 selectively inhibits Rpb3-high-expression HCC cells proliferation, migration and tumorigenesis **(A)** Ad-Rpb3-N1 infection decreased proliferation of HCC-LM3 cells. **(B)** Ad-Rpb3-N1 infection inhibited migratory ability of HCC-LM3 cells. **(C)** Average tumor volume in athymic nude mice subcutaneously inoculated with HCC-LM3/Ad-V and HCC-LM3/Ad-Rpb3-N1. **(D)** The number of tumors counted from the surface of liver lobes. **(E)** Tumor size measured on the surface of liver lobes. For D and E, C57BL/6 mice treated with 50 μg/g of DEN at age 20 days and killed 9 months later. **(F)** Rpb3-N1 did not affect endogenous Rpb3 binding to Rpb11. Endogenous Rpb11 was immunoprecipitated from the L02 cell lysates using rabbit anti-Rpb11 antibody, followed by immunoblotting with antibodies to Rpb11 and Rpb3. Sample loading controls are shown (2% input). **(G)** Quantitative ChIP analysis of RNA Pol II enrichment on selected genes using L02 cells. Immunoprecipitations were performed using antibodies against CTD (8WG16) for the RNA Pol II Rpb1 subunit. Immunoprecipitated fragments from ChIP experiments were amplified with primers as indicated in the Method and Material section. Human genes *ADH1*, *RPL28*, *RPL17*, and *ACT1* were detected, yeast gene *GAL1* was used as a system non-transcribed negative control. No CHIP signals for *GAL1* were detected in our system. Error bars represent the standard deviation between at least three biological replicates. **(H)** q-RT-PCR analysis for mRNA level of selected RNA Pol II transcribed genes. **(I)** Rpb3-N1 did not inhibit normal liver cell line L02 proliferation. **(J, K)** Rpb3-N1 did not inhibit Rpb3 low-expression cell line QGY-7701(J) and HepG2 (K) cells proliferation. Results represent at least three separate experiments. n=15/group (C-E). Error bar represent ± S.D. * *p* < 0.05, *** *p* < 0.001.

To investigate further the role of Rpb3 in liver tumorigenesis, DEN-induced liver cancer model was used. We injected 50 μg/g DEN into C57BL/6 mice and found that Rpb3 expression was up-regulated in DEN-induced tumor tissues, compared with liver tissues from PBS treated mice (Supplemental Figure S4 A, B). We injected 50 μg/g DEN into C57BL/6 mice and treated these mice with Ad-V or Ad-Rpb3-N1 once a week. The expression of Rbp3-N1 was shown after adenovirus infection (Supplemental Figure S4 C, D). After 9 months, both the number and size of liver tumors in mice treated with Ad-Rpb3-N1 were decreased compared to mice treated with Ad-V (Fig. 5D and 5E). These results indicate that C-terminus of Rpb3 could inhibit liver tumorigenesis.

### The RNA Pol II activity is not changed in HCC tumor samples and HCC cell lines

Since only Rpb3 was up-regulated in HCC, while the expression of all the other 11 subunits of RNA Pol II was not changed (Supplemental Fig. S1 and S2), we thus suspected that the enhanced HCC staging and HCC cell proliferation induced by Rpb3 might be not due to the RNA Pol II activity changing. To verify our hypothesis, we used CHIP assay to detect the association between RNA Pol II and a set of selected Pol II-transcribed genes [14, 15], Human genes *ADH1*, *RPL28*, *RPL17*, and *ACT1* were detected here, yeast gene *GAL1* was used as a system non-transcribed negative control. No changes were observed in different tumor stages (Supplemental Fig. S5A). The mRNA level of all these selected RNA Pol II-transcribed genes in different HCC stage was not changed either (Supplemental Fig. S5B). We observed the similar results in HCC cell lines. RNA Pol II bound similar level of selected RNA Pol II-transcribed genes, no matter the cells expressed high or low Rpb3 (Supplemental Fig. S5C), and the mRNA level of these selected Pol II-transcribed genes in different HCC cell lines is similar too (Supplemental Fig. S5D). To demonstrate our CHIP assay system for RNA Pol II binding to selected RNA Pol II-transcribed genes working well, we used Med 17 as our system positive control [14]. When we transfected Med17 into HepG2 cells, we observed enhanced binding between RNA Pol II and selected RNA Pol II-transcribed genes (Supplemental Fig. S5E). To demonstrate the qRT-PCR assay system for detecting selected RNA Pol II-transcribed genes working well, we transfect the plasmids of selected RNA Pol II-transcribed genes to HepG2 cells and observed enhanced mRNA level of these genes (Supplemental Fig. S5F).

### N-terminus of Rpb3 does not inhibit normal liver cell and Rpb3 low-expression HCC cell proliferation

Since Rpb3 is one of subunits of RNA polymerase II and binds directly to Rpb11 [16-18], we suspected whether Rpb3-N1 destroyed RNA polymerase II complex by blocking Rpb3/Rpb11 association. Using co-IP assay, we found that Rpb3-N1 did not bind to Rpb11 (data not shown), nor inhibited endogenous Rpb3 binding to Rpb11 (Fig. 5F). Using quantitative ChIP analysis, we found that RNA Pol II enrichment on selected genes was not inhibited by Rpb3-N1, while knockdown of Rpb3 through Rpb3-shRNA decreased RNA Pol II enrichment on selected genes (Fig. 5G). The mRNA level of selected RNA Pol II-transcribed genes was not decreased by Rpb3-N1 either (Fig. 5H).

For function study, we infected normal immortalized hepatocyte cell line L02, Rpb3-low-expression HCC cell lines QGY-7701 and HepG2 with Ad-Rpb3-N1, and established stable cell lines individually. Using MTT and BrdU cell proliferation assay, we found that Rpb3-N1 did not inhibit normal liver cell line L02 proliferation (Fig. 5I). These results indicated that Rpb3-N1 did not block regular RNA polymerase II function. HCC cell lines QGY7701 and HepG2 cells expressed similar Rpb3 protein level and mRNA level as normal liver (see Figure Supplemental Figure S2, A and B). To our surprise, Rpb3-N1 did not inhibit QGY7701 and HepG2 cells proliferation (Fig. 5G and 5K). These results suggested that Rpb3-N1 selectively inhibited Rpb3-high-expression HCC cells proliferation, but not inhibited normal liver cells and Rpb3-low-expression HCC cells proliferation.

### Snail knockdown inhibits Rpb3 induced HCC cell proliferation and migration

We next tested whether Snail is necessary in Rpb3 induced HCC cells proliferation, migration and tumor growth. Using shRNA, we knocked down endogenous Snail in Rpb3-overexpressing QGY-7701 cells and HepG2 cells (Supplemental Figure S6A) and found (using the MTT assay) that knockdown of Snail inhibited HCC cell proliferation *in vitro* (Supplemental Figure S6B and C). Also, the migration of Rpb3-overexpressing QGY-7701cells and HepG2 cells were inhibited by knockdown of Snail (Supplemental Figure S6, D and E). Furthermore, the *in vivo* tumor growth was dramatically inhibited by Snail shRNA compared with control shRNA (Ctrl shRNA) both in Rpb3-overexpressing QGY-7701 cells and HepG2 cells (Supplemental Figure S6, F and G). These results demonstrated that Snail is necessary in HCC cell proliferation and migration induced by Rpb3.

## DISCUSSION

In this study, we showed that Rpb3 expression is frequently up-regulated in HCC (51.24%), particularly in advanced stage of HCC (Stage IV, 72.63%), and there was a positive correlation between Rpb3 expression and advanced clinicopatological features. In addition, the Rpb3 expression correlated with poor overall and disease-free survival in patients diagnosed with HCC. Functional analysis through gain- or loss-of-function studies showed that Rpb3-overexpression enhanced HCC cell proliferation, migration and *in vivo* tumor growth, whereas Rpb3-knockdown using shRNA inhibited HCC cell proliferation, migration and *in vivo* tumor growth. These results suggested that Rpb3 is critical regulator of hepatocyte proliferation during tumorigenesis and liver regeneration.

Rpb3 is a core subunit of RNA polymerase II, which is a central enzyme required for the transcription of essentially all pre-mRNAs in eukaryotic cells. Rpb3/Rpb11 form a heterodimer that is considered as the functional counterpart of the bacterial α subunit involved in promoter recognition [16-18] and also plays a central role in the interaction between RNA polymerase II and the mediator complex [14, 19]. In addition to its essential structural function in RNA polymerase II, RPB3 display an active role in tissue-specific transcription. For example, Rpb3 directly contacts the myogenic transcription factor Myogenin[6] and the activating transcription factor ATF4 [7]. Other subunits of RNA Pol II, Rpb5 [20-22], Rpb7 [23] and Rpb2/Rpb10α [24], also were involved in specific transcription regulation. However, no studies were reported the roles of RNA polymerase subunits in cancer development. To our knowledge, for the first time, we showed that overexpression of Rpb3 played as an oncogene in HCC progress. The most interesting thing is that it seemed Rpb3 promoted HCC cell proliferation not through regulating RNA Pol II function, for no other subunits of RNA Pol II were observed up-regulated in patients diagnosed with HCC, and the function of RNA Pol II did not changed along with Rpb3 expression in HCC cells either. Using this mechanism, we created adenovirus coding N-terminus of Rpb3 and found that the first 50 amino acids of Rpb3 blocked Rpb3/Snail association, but not blocked Rpb3/Rpb11 association or RNA Pol II function. Particularly, Rpb3-N1 selectively inhibited Rpb3-high-expression HCC cells proliferation but not inhibited normal liver cells proliferation and Rpb3-low-expression HCC cells proliferation. Our results strongly indicated that there are at least two roles of Rpb3 in cell proliferation: 1) regular expression level of Rpb3 contributes its function to RNA polymerase II complex for regular cells survive; 2) enhanced expression of Rpb3 in HCC progress contributes its function in the ways beyond RNA polymerase II complex. For example, binding to Snail here in our study is one of the ways. It would be very interesting to study the various functions and mechanisms of Rpb3 in various conditions.

The most advantage in our study is that Rpb3-N1 selectively inhibited Rpb3-high-expression HCC cells proliferation, but not inhibited normal liver cells proliferation. Rpb3-N1 thus could be as perfect medicine target with low side effect. Patients diagnosed with Rpb3-high-expression HCC could be considered selectively to be treated with these antagonists.

## METHODS

### Patients and immunohistvochemical staining

HCC tumorous and adjacent nontumorous liver tissues were collected from 322 patients who underwent curative surgery for HCC at Taizhou Hospital of Zhejiang Province and Eastern Hepatobiliary Surgery Hospital. Informed consent was obtained from each patient, and the study protocol was approved by the Clinical Research Ethics Committee of Wenzhou Medical University and Second Military Medical University. A diagnosis of HCC was confirmed on histologic examination. Tumor stage was classified according to American Joint Committee on Cancer criteria.

Immunohistochemical staining was performed as previous.[25-27] For the determination of Rpb3 immunoreactivity cytosolic or nuclear staining of the yellowish or brownish granules was graded using the following scale: 0 for background staining, 1 for faint staining, 2 for moderate staining and 3 for strong staining. The intensity was judged relative to HepG2/Rpb3 cells which also served as staining positive controls and was arbitrarily designated as 3. In addition, positive cells number expressed as percentages of total cells number throughout the entire tissue section were graded according to the following scale: 0 for < 5%, 1 for 5-25%, 2 for 26-50%, 3 for 50-75% and 4 for 75%-100%. When combining these two parameters, staining intensity and the percentage of positivity of tumor cells were multiplied to produce a weighted score for each tumor specimen. 0-2 and ≥ 3 were considered negative and positive staining, respectively.

### Cell cultures, plasmids and antibodies

HCC cell lines HepG2, Hep3B, HCC-LM3, SMMC-7721, QGY-7701, and BEL-7402, were purchased from American Type Culture Collection (ATCC). Normal human liver cell line L02 was obstained from China Center for Type Culture Collection (Shanghai). The cells were cultured according to the recommendations from ATCC. QGY-7701 and HepG2 cells were transfected with the plasmids of full-length, wild-type Rpb3 or the plain vector, HCC-LM3 and SMMC-7721 were transfected with the plasmids of Rpb3 shRNA or control shRNA, using Lipofectamine 2000 (Invitrogen). The positive transfectants were selected using 0.8 mg/ml G418 (GIBCO BRL) for two weeks, to obtain stable cells pool for overexpression or knockdown of Rpb3 for using in subsequent assays. For adenovirus infected cells, 1X10^8^ pfu adenovirus containing according construction was used to infect cells, 0.8 mg/ml G418 was used to select for two weeks, to obtain according stable cells pool for using in subsequent assays.

Human Rpb3 shRNA1, target sequences: 5′-TTATTAACAGCAGTCAGGG -3′, human Rpb3 shRNA2 target sequence: 5′-TCATTGCACCGCACATCGA -3′, and none sense shRNA control target sequence: 5′-TGAGCAGGCGCATGTGCTG-3′, Human Snail shRNA, target sequences: 5′-TAATATTCAAGGCTCGGAG -3′, all the shRNA plasmids were obtained from Thermo Scientific (U.S.). The plasmid of Rpb3 (MHS6278-202801899) and Snail (MHS6278-202758251) were purchased from Thermo Scientific. Primary antibodies to Rpb3, Snail, Rpb11 were purchased from Abcam. Primary antibodies to β-actin, GST-Tag, His-Tag and Flag-Tag were purchased from Sigma. Second antibodies anti-mouse IgG-HRP and anti-rabbit IgGHRP were purchased from Sigma. MTT assay reagents were purchased from DingGuo Biotech.

### Real-time qPCR

Real-time qPCR (qRT-PCR) assay was performed as previous [25, 26]. Total RNA was extracted using the Absolutely RNA Miniprep Kit (Stratagene) and reverse transcribed using ThermoScript RT-PCR System (Invitrogen). The resulting cDNA was used for real-timePCR using the SYBR-Green Master PCR Mix (Applied Biosystems) in triplicates. All RT^2^ qPCR Primer pairs were purchased from SABiosciences. PCR and data collection were performed using the Mx3000 qPCR System (Stratagene). All quantitations were normalized to an endogenous β-actin control. The relative quantitation value for each target gene was compared with the calibrator (β-actin), which was expressed as 2^−(Ct-Cc)^ (Ct and Cc are the mean threshold cycle differences after normalizing to β-actin). The Primers for qRT-PCR: Rpb1 Forward: catgcccgctgcgcaccatc; Rpb1 Reverse: aatgtggccaaagtggccag; Rpb2 Forward: atgatgatgaaatcaccccg, Rpb2 Reverse: cttcattgggcatcattggt; Rpb3 Forward: accaatgatgcccaatgaag; Rpb3 Reverse: agatgaggtctcgagacgtg; Rpb4 Forward: agcgatccgcgggctggcga; Rpb4 Reverse: aggccaactcaaacttatga; Rpb5 Forward: tggaaaatcc gcaagaccat; Rpb5 Reverse: tgcaccacgatgagagcccg; Rpb6 Forward: gacgactttgatgatgtgga; Rpb6 Reverse: ttcctcctacttcctggtga; Rpb7 Forward: atatctccctagagcacgaa; Rpb7 Reverse: ggatggaatgtcgagagatg; Rpb8 Forward: gatctaatcttagatgtaaa; Rpb8 Reverse: ctagcttcttcatcaggaga; Rpb9 Forward: gggacttacg agccgggctt

Rpb9 Reverse: tgccgcggac cgaggaccac; RPb10 Forward: cctgtacgctgcttcacttg; Rpb10 Reverse: tctccaggggtgcataattg; Rpb11 Forward: gggcgagaagaagatcacca; Rpb11 Reverse: cacccgaaagcgctcctcca; Rpb12 Forward: aaggacgttcaacctccaaa; Rpb12 Reverse: gagcatcaaaaacgaccaat; β-actin Forward: aagaagagatcgccgcgctg; β-actin Reverse: cgcagctcgttgtagaaggt.

### CHIP

CHIP experiments were performed as described [15]. Cells were cross-linked with 1% formaldehyde for 10 min. Pol II was immunoprecipitated with 8WG16 anti-CTD antibody (Covance), and bound to IgG magnetic beads (Dynabead). Immune complexes were washed. Immunoprecipitated DNA was analyzed by quantitative real-time PCR on an ABI Prism 7000 or 7300 machine (Applied Biosystems). Relative quantification using a standard curve method was performed and the occupancy level for a specific fragment was defined as the ratio of immunoprecipitated DNA over total DNA. Human genes *ADH1*, *RPL28*, *RPL17*, and *ACT1* were detected, yeast gene *GAL1* was used as a system non-transcribed negative control. No CHIP signals for *GAL1* were detected in our system. The Primers for real-time qPCR are, ADH1 Forward: GAGTTCCTAAGAAATTTCCT; ADH1 Reverse: GTCTCCTGCATCTATCTCAA; RPL28 Forward: GAAAACTTCCGAACGGTTCC; RPL28 Reverse: CCGAGGCGGCTCGATGT; RPL17 Forward: AAGACAGGTGAAAGGGTTGC; RPL17 Reverse: TAGTTGCTCGGTTTTGTTTG; ACT1 Forward: TGGTTCATTAAGAAGAAACA; ACT1 Reverse: TTACCCCAGCTGCTTCGTCA; GAL1 Forward: AAAGAAACTTGCACCGGAAA; GAL1 Reverse: GGCCCATATTCGCTTTAACA.

### Liver cell isolation for qRT-PCR and western blotting analysis

Liver cells were isolated using a standard three-step protocol. Liver perfusion was initiated by administering through the portal vein 200 ml of 0.5 M EGTA solution in basic liver perfusion buffer (30 mM KCl, 1.3 M NaCl, 10 mM NaH2PO4.2H2O, 100 mM Glucose and 100 mM HEPES, pH7.4). The liver was then washed with 200 ml of basic liver perfusion buffer alone. Subsequently, 0.02% collagenase type 4 (Sigma-Aldrich) and 5 mM CaCl2 were added to the basic liver perfusion buffer and perfusion was continued until digestion was complete. The digested liver was suspended in 50 ml of PBS and the dissociated cells were passed through a 100 μm nylon mesh and centrifuged at 50 g for 5 minutes at 4 °C. After centrifugation, precipitated cells were used as hepatocyte fraction. Hepatocytes were identified as large (20–25 mm), frequently binucleate cells with basophilic cytoplasm. The preparation was less than 5% contaminated by other cell types. Cells were washed three times in Williams media, and viability was checked by trypan blue exclusion. Isolated hepatocytes were then analyzed by qRT-PCR and western blotting assay for detecting mRNA level and protein level of Rpb3.

### Adenovirus tail vein injection for intrahepatic expression of Rpb3, Rpb3 shRNA, and Snail mutants

The forward primer 5′-AATCTAGAATGCCGTACGCCAACCAGCCTACC-3′ and the reverse primer 5′-ACAAGCTTTCACTTTCGAGCCTGGAGATCCTTGG-3′ were used to amplify N-terminus of Rpb3 which was then digested with Xba1/HindIII and ligated into the vector of DUALGFP-CCM for Ad-Rpb3-N1 construction. The construct was verified by DNA sequence analysis. All the proteins were fused with a Flag tag and the expression of them were detected using anti-Flag antibody (Sigma). The high titers of custom-made Ad-Rpb3N1 and its control adenoviral vector (Ad-V) were purchased from Vector Biolabs (US). 1X10^8^ pfu adenovirus containing accordingly construction was injected into tail vein mouse. Liver samples were obtained at 0, 1, 2, 3, 4, 5, 6, 7 for Rpb3 protein detecting after liver cell isolation by western blotting.

### DEN-induced hepatocarcinogenesis and Tissue Collection

Male C57BL/6 mice were given at postnatal day 20 a single intraperitoneal injection of DEN (50 μg/g body weight). One week after DEN treatment, the DEN-challenged mice were given intraperitoneal injections of Ad-GFP or Ad-Rpb3-N1 (1X10^8^ pfu) once every week until killing and necropsy at 9 months. The livers were then separated into individual lobes, analyzed for tumors number and tumor size.

### Immunoblotting and immunoprecipitation assay

Cells were lysed with ice-cold radioimmunoprecipitation assay lysis buffer at 4°C for 1 hrs. Samples were subjected to SDS-PAGE, transferred to PVDF membranes (Millipore) and detected using appropriate primary antibodies followed by horseradish peroxidase-conjugated goat anti-mouse or rabbit IgG. The blotting signals were detected using SuperSignal West Dura Extended Duration Substrate (Pierce).

For immunoprecipitation, 1 μg appropriate antibody was preincubated with 30 μl slurry of Protein A-agarose beads (GE Healthcare Life Sciences). Lysates (~1 mg/sample) were incubated with the antibody-bound Protein A-agarose beads at 4°C overnight. After extensive washing with the radioimmunoprecipitation assay lysis buffer, samples were resuspended in the reducing SDS sample loading buffer, boiled for 5 min, and subjected to SDS-PAGE and immunoblotting.

### Cell Proliferation

For MTT assay, the cells, including all transfectants, were grown to the exponential phase and detached through trypsin treatment. Viable cells (5 × 10^3^ cells/ml) were plated onto 96-well tissue culture plates (100 μl complete medium/well) and cultured at 37°C in 5% CO_2_. At different time points, tetrazolium salt was added (20 μl per well) and incubated at 37°C for 4 hr. The insoluble blue formazan product was solubilized by addition of 100 μl/well 10% SDS/5% isobutanol. The plates were read on a micro-titer plate reader using a test wavelength of 570 nm and a reference wavelength of 630 nm [25].

For the BrdU assay, 1.5x10^5^ cells/ml were seeded into a 35-mm dish. After one day, 0.4% FCS was used to arrest cells at the G0 phase. After two days, BrdU (30 mg/l) was added to the cells for 40 min. After washing three times with PBS, the cells were fixed using methanol for 10 min and 0.3% H2O2 for 30 min. A 5% BSA solution was used to block for 1 h followed by treatment with famide at 100°C for 5 min. After washing with PBS, anti-BrdU antibody was added to the cells. The color was subsequently developed through incubation with the ImmunoPure Metal Enhanced Diaminobenzidine (DAB) Substrate kit (Pierce). The number of BrdU-positive cells and total cell number were counted.

### Boyden chamber migration assay

The cell migration assay was conducted in a 48-well micro-chemotaxis chamber (Neuro Probe, Inc.). PVP-free polycarbonate membranes (8 μm pores) were coated with 1% gelatin. The bottom chambers were loaded with medium with 5% FBS while the upper chambers were seeded with HCC cells (5x10^5^ cells/ml), resuspended in medium with 1% FBS. They were incubated at 37^o^C for 6 hr. The filters were then fixed, stained with 0.5% crystal violet, and the cells that had migrated through the filters were counted [25].

### Nude mice tumor growth

Stable cell lines (pool), QGY-7701/V, HepG2/V, QGY/Rpb3, HepG2/Rpb3, HCC-LM3/control shRNA, SMMC-7721/control shRNA, HCC-LM3/Rpb3 shRNA1, HCC-LM3/Rpb3 shRNA1, SMMC-7721/Rpb3 shRNA1 and SMMC-7721/Rpb3 shRNA2, were re-suspended at 5 × 10^7^ cells/ml and a 0.1-ml aliquot of cell suspension was injected subcutaneously into athymic nude mice (*n* = 10/group). The tumor volume was measured at different time points. The tumor volumes were determined through external measurements and calculated according to the equation, V = [L × W^2^] × 0.52 (V = volume, L = length, and W = width). The data were analyzed using Student's *t*-test, and *p* < 0.05 was considered significant [25].

### Statistical analysis

The overall survival is represented in months, defined as the interval between the date of the surgery and the date of death or last follow-up. Overall survival curves were estimated using the Kaplan–Meier method, and the difference in survival was evaluated using the log-rank test. The *p* values of less than 0.05 and 0.01 were considered statistically significant and very significant, respectively. All computations were performed using R 2.9.0 software (www.r-project.org).

### Ethics Statement

For all animal involving study, the study protocol was approved by the Clinical Research Ethics Committee of Wenzhou Medical University and Second Military Medical University. And our policy is consistent to The U.S. Public Health Service *Policy on Humane Care and Use of Laboratory Animals*, available from the Office of Laboratory Animal Welfare, National Institutes of Health, Department of Health and Human Services.

Supplemental Tables, Supplemental figures and methods are available in online **Supplemental Material**

## SUPPLEMENTARY MATERIALS FIGURES AND TABLES


